The article "Analysis of Sports Knee Fractures Based on X-Ray and Computed Tomography Imaging" was published in 2021. Journal: Comput Math Methods Med.

# Analysis of Sports Knee Fractures Based on X-Ray and Computed Tomography Imaging

**DOI:** 10.1155/2021/9572363

**Published:** 2021-12-01

**Authors:** Bo Cui, Yan Liu, Shuxiang Chen

**Affiliations:** ^1^Jiangmen Polytechnic, Jiangmen Guangdong 529000, China; ^2^Department of Orthopaedic Surgery, Jiangmen TCM Affiliated Hospital of Jinan University, Jiangmen Guangdong 529000, China

## Abstract

**Objective:**

To analyse the X-ray and computed tomography (CT) findings of 128 patients with sports-related knee fractures and to improve the diagnosis rate based on the existing methods of diagnosis of sports knee fractures on X-ray and CT images.

**Method:**

In this study, we retrospectively analyse the medical records of 128 cases of sports-related fractures in the hospital, analyse the results of X-ray examination and CT imaging of patients with sports knee fractures, and compare the results obtained by the two examination methods, while referring to MRI images performed.

**Results:**

CT examination of knee fractures, tibial plateau fractures, and knee joint free body results were compared with X-ray results (*P* < 0.05), while CT examination of patella fractures and X-ray results were compared. The difference was not statistically significant (*P* > 0.05).

**Conclusion:**

For imaging examination of knee fractures, a single ordinary X-ray or CT scan should be selected according to the specific situation of the patient. For patients with suspected unstable fractures, when the patient's informed consent and the condition are not allowed, ordinary X-ray film combined with CT examination is used to improve the accuracy of diagnosis and avoid the existence of hidden fractures, resulting in medical accidents.

## 1. Introduction

With the continuous improvement of the quality of life, people are very easy to fall their knees in pursuit of extreme sports. At the same time, they are industrialized. When people produce labor sports, they are very easy to be injured by mechanical facilities [1]. Therefore, in recent years sports knees the share of fractures in bone and joint trauma continues to rise, and there are currently certain loopholes in the way of examination of sports knee joints, which leads to the patient's invisible fracture site not being treated in time, causing permanent injury to the patient's fracture site and actual inspection at the fracture site. In the middle and knee fractures, due to the very complicated anatomical structure, clinical diagnosis cannot be made in time, and it is easy to cause missed diagnosis, and there is a hidden danger of medical treatment accidents [2]. At present, there are two main diagnostic techniques for diagnosing sports knee fractures, which are X-ray examination and CT imaging examination.

X-ray examination and CT imaging examination as the main means of sports knee fracture are widely used in clinical practice. Upon application, these two examination techniques have certain advantages and disadvantages [3]. The advantages of X-ray examination are as follows: good diagnostic value for displaced fractures and opaque foreign body retention and finding that the patient is changing position fractures that can only be felt at the time. The disadvantages of X-ray examination are as follows: radiation is harmful to the human body, so it is not suitable for pregnant women and other special populations. X-ray examination still has unclear tissue imaging and poor contrast and cannot identify fine structures. The advantages of CT imaging examination are as follows: high-density tissue imaging is clear, and the accuracy of measuring the distance between bone structures is high [4].

Multirow spiral CT can carry out three-dimensional imaging, which is helpful to display tissue and organ lesions in three dimensions. The disadvantage of CT imaging examination is as follows: CT scanning is limited to the technical level of technical personnel. The interval limit of the scanning plane cannot correctly read the information of the examination site, resulting in a certain rate of missed diagnosis. CT has low definition and resolution of soft tissue imaging [5]. Due to radiation problems, pregnant women and special populations cannot use it. Because of these advantages and disadvantages, these two inspection techniques often have different detection results at different fracture sites, and there are certain inspection loopholes. The inspection results are inaccurate, which is likely to cause medical accidents during treatment and cause secondary injuries to patients.

Therefore, in order to reduce the loopholes in the examination of sports knee fractures in the future, this article retrospectively analysed the results of X-ray examination and CT examination of 128 sports knee fractures archived in the hospital medical record using *χ*^2^ test and compared them [6]. The *χ*^2^ test is mainly used to calculate the two attributes of two or more sets of data and the comparison between two or more phenomena. For example, to test the difference between the two sampling rates and the composition ratio, *χ*^2^ is a kind of a simple and widely used difference significance test method, which can better compare the results of X-ray examination and CT examination of 128 cases of sports knee fractures and compare them. The following is our detailed experimental method. The implementation of multilayer spiral computed tomography (MSCT) scanning and three-dimensional reconstruction technology for patients with extremity bone and joint fractures can help to quickly and accurately diagnose the damage of extremities and joints [6–9] and provide more detailed imaging data for the clinical treatment of patients. The effective use of multislice spiral CT postprocessing technology can establish three-dimensional images and intuitively feedback the images of the patient's limbs and joint fractures.

## 2. Methods and Materials

### 2.1. General Materials

A total of 128 patients with sports knee fractures in the hospital were selected as the research object, including 76 males and 52 females, aged 14 to 69 years, with an average age of 38.64 ± 5.33 years. The time of consultation after injury was <24 h (56 cases) (43.75%), 24 h ~72 h (60 cases) (46.88%), and >72 h (12 cases) (9.38%); injured part: 48 cases (37.50%) of left knee joint injury, 50 cases of right knee joint injury cases (39.07%), and 30 cases of knee injury (23.44%); fracture causes: 69 cases of traffic injuries (53.91%), 22 cases of sports (17.09%), 20 cases of falls (15.63%), 17 cases of high-level fall injuries (13.28%); 21 cases (16.44%) with other site fractures, 13 cases (10.16%) of chest trauma, 9 cases (7.03%) of abdominal organ injuries, and 3 cases (2.34%) of craniocerebral injury; 128 patients: 54 cases (42.19%) with mid-knee pain, 24 cases (18.75%) with swelling, 19 cases (14.84%) with knee interlocking, and 11 cases (8.59%) with dysfunction; and 128 patients having positive lateral compression test: 43 cases (33.59%) and 23 cases positive for drawer test (17.97%).

### 2.2. Inspection Method

In all cases, routine and special X-ray plain film examinations are performed at the time of treatment after injury to observe the knee joint injury, whether there are suspicious fractures or hidden fractures. The CT examination was completed within 7 days after the injury, and all cases were examined using the Toshiba Activation 16TSX-031A multislice spiral CT machine [7]. The patient was lying on his back, with his feet advanced. The scanning range was determined by X-ray film. The scanning conditions were 120 kV, 200 mA, 3 mm layer thickness, 3 mm interval, and 512 × 512 array. When a meniscus fracture is suspected, a 1 mm continuous thin-layer scan is used. The scanning slice is as parallel as possible to the knee joint surface. The scanning range includes the proximal tibia and the distal femur [8]. Bone window was used to observe the fracture, and soft tissue window was used to observe the damage of soft tissue, ligament, and meniscus. Coronal and sagittal images were reconstructed and assisted with cutting techniques for the cases of tibial plateau collapse, tibial plateau fracture fragment displacement, meniscus injury, and dislocation of the knee joint, and each bone end making up the knee joint was observed separately [9].

### 2.3. Statistical Methods

The *χ*^2^ test is a widely used, simple, and commonly used difference significance test method. It can be mainly used to count the two types of attributes of two or more groups of data and the comparison between two or more types of phenomena, such as testing the difference between two sample rates and composition ratios [10–13].

Basic principles and steps are as follows: the basic principle of the *χ*^2^ test is to assume that each sample comes from the same attribute of the population; the difference between the actual data in each group is only due to sampling error; by calculating the discrete situation of the actual number and the theoretical number of each group, the total error is obtained *χ*^2^ value, so as to determine the probability of the existence of the hypothesis, that is, the probability *P*. If the hypothesis is true, then, the *χ*^2^ value will not be very large, but keep it within a certain range, the corresponding *P* value is greater than 5% (*P* > 0.05); that is, the probability of such a large difference between samples due to sampling errors alone is greater than 5%, indicating that there is no obvious difference between the samples in essence. They come from the population of the same attribute, and the assumption is affirmed. In other words, if the calculated *χ*^2^ value is large and exceeds a certain range, the corresponding *P* value is less than 5% or 1%; that is, the probability of such a large difference between samples due to sampling errors is less than 5% or 1%; indicating that the difference between the groups is not due to sampling, there may be a difference between the two, they are not from the same attribute of the population, and the assumption is rejected [14].

## 3. Results

X-ray showed that the fracture was located on the posterior side of the medial condyle of the tibia. No abnormal findings were found on the DR examination film. Ten cases showed a localized compact line on the posterior side of the medial condyle of the tibia (Figure 1(a)). 21 cases of fractures located on the posterior side of the middle and upper tibia and the posterior side of the middle tibia had no abnormal findings on DR film; 19 cases showed bone injury reaction, 18 cases were laminar, 12 cases were mound-like, and 9 cases were marginal smooth. Five cases had uneven edges (Figure 2). If the fracture was located in the lower tibia, there were no abnormal findings in 2 cases of DR film, and 2 cases showed oblique dense lines. If the fracture is located on the outer posterior side of the lower femur, the DR film shows the reaction of the laminar bone injury on the outer posterior side, and the local bone density increases. The fractures were located in the middle and distal segment of the second metatarsal bone. In 4 cases, the bone injury reaction was seen, which was layered or mound-like, and the edges were smooth; 1 case had a thickened cortex and local hemispherical bulge, which was shaped like a button, and showed a “button sign” (Figure 3).

### 3.1. CT Manifestations

Among the CT-examined patients, 28 cases had no abnormal findings; 13 cases showed fracture lines, of which 8 cases were translucent lines and 5 cases were high-density lines; 15 cases showed periosteal reaction, of which 13 cases showed periosteal hyperplasia surrounding the cortical bone, a “double cortical sign”; 13 cases of local cortical thinning, blurred edges, showed a “gray cortical sign” as shown by (Figure 4(a)); 11 cases around the fracture line around the bone cortical periosteum reaction was partially interrupted, shaped like a navel, manifested as “umbilical concave sign,” of which 7 cases showed double “umbilical concave sign” (Figure 4); 14 cases showed bone callus formation and increased bone marrow cavity density; 6 cases showed thickening of the cortical bone and smooth border; 9 examples show swelling of soft tissue.

Compared with the performance of reference MRI in fracture examination, patients with MRI examination all found positive findings, which were characterized by sharp line-like low-sign fracture lines on the edges of T1WI and T2WI and long T2 bone marrow enema signal; the border is unclear; STIR sequence showed a significant high signal (Figure 1(a)). 17 cases showed different degrees of soft tissue enema.

CT examination of floating knee fractures, tibial plateau fractures, and knee free body results were statistically significant compared with X-ray results (*P* < 0.05); while CT examination of patella fractures was compared with X-ray results, the difference was not statistically significant (academic significance: *P* > 0.05). The data can be depicted by Table 1.

## 4. Discussion

Current imaging methods for sports knee fractures include general X-ray, CT, MRI, and radiation computed tomography (ECT). In the clinical examination of sports knee fractures, X-ray positive photography is the preferred method of examination, but it can only show the structure of the knee joint from the front-back direction and the left-right direction and can only provide the general shape of the bone. Online examinations are usually negative. Usually, it takes 2 to 3 weeks from the patient's symptoms to the positive signs of plain X-ray film [15].

Understanding the mechanical structures of the bones via medical imaging can allow us to comprehend the involved structural mechanics and help to understand fractures. For occult trabecular fractures and occult fractures, it can be seen that the local bone density exhibits uneven imaging characteristics. Because the front and back bones or left and right bones on the X-ray film overlap, it is impossible to clearly show the state of small fracture line tearing, traveling, or displaced bone fragments, and at the same time, it is impossible to show bone contusion, meniscus, and ligament damage. It is easy to miss the diagnosis.

Clinical diagnosis cannot provide accurate information. CT examination can obtain a clearer tomographic image, which is a more advanced examination method, which can accurately display the existence of avulsion fracture and its avulsion site, solve the problem of overlapping images, and display the fracture line more clearly [16]. There are changes in walking, location, type, degree of displacement, range, and surrounding soft tissue; however, its disadvantage is that it shows some concave lesions in the direction of the long axis, and it is impossible to analyse the changes of the fracture as a whole. The results showed that the detection rate of 128 cases of knee fractures by X-ray examination was 84.37%, which was 99.22% lower than the detection rate of CT examination, suggesting that CT examination has higher accuracy in diagnosis of sports knee fracture. CT three-dimensional reconstruction technology can better observe the internal condition of the patient's joints and avoid the limitations of plain X-ray diagnosis.

The results showed that patients with knee fractures could not be diagnosed only by X-ray examination, which could not fully reflect the actual situation of sports knee injury, and the examination results could only be used as a diagnostic reference. Therefore, after X-ray examination of patients in the clinic, CT and 3D reconstruction techniques should be used to improve the accuracy of diagnosis and avoid misdiagnosis and misdiagnosis of X-ray examination of patients. The three-dimensional effects of SSD and VRT are obvious [14–16]. Because SSD adopts threshold imaging, it is suitable for the display of the surface morphology of the skeletal system. It has a strong spatial three-dimensional effect and a clear surface anatomy relationship, which is conducive to the positioning of the fracture and the extent of the fracture line. The performance is obviously affected by the segmentation threshold in image processing, so the internal structure of the object cannot be displayed, and the density information of the object [17] cannot be provided. Orthopedic imaging can use deep learning for diagnosis [18].

## 5. Conclusion

In summary, in order to improve the diagnostic accuracy of sports knee fractures, when patients undergo X-ray or CT imaging tests, patients should be encouraged to undergo plain X-ray examinations, and CT examinations should be considered according to the patient's condition. For patients with suspected unstable fractures, if the patient's permission is given and the patient's condition is informed, ordinary X-ray film combined with CT examination can be used to improve the accuracy of diagnosis, avoid hidden fractures, and cause harm to the patient's body, including psychology, which can ensure the accuracy of the test to the greatest extent and the effectiveness of the later treatment.

## Figures and Tables

**Figure 1:** Stress fracture associated with tibial condyle motion based on (a) DR-positive film and (b) MRI coronal radiograph.

**Figure 2:** Patient's upper tibial motion fracture based on (a) DR-positive film and (b) DR side slice.

**Figure 3:** Patient's metatarsal motion fracture.

**Figure 4:** The patient's middle and upper tibial motion fracture image diagnosis based on CT cross-section slice and (b) CT cross-section slice.

**Table 1:** The results of X-ray and CT examination for the diagnosis of knee fracture.

Type of fracture	Number of cases	X-ray inspection results	CT examination results	*χ* ^2^	*P*
Floating knee fracture	50	42 (84.00)	49 (98.00)	5.98 < 0.05	
Type I bicondylar fracture	18	16 (88.89)	18 (100.00)		
Type II backbone fracture	20	17 (85.00)	20 (100.00)		
Type III is mixed	12	9 (75.00)	11 (91.67)		

Tibial plateau fracture	68	56 (82.35)	68 (100.00)	13.16 < 0.01	
Simple tibial lateral epicondyle split fracture	10	7 (70.00)	10 (100.00)		
Lateral epicondylar split fracture combined with platform	8	4 (50.00)	8 (100.00)		
Collapse fracture					
Simple platform central collapse fracture	7	4 (57.14)	7 (100.00)		
Medial platform fracture	12	10 (83.33)	12 (100.00)		
Fracture of medial and lateral epicondyle of tibia	13	13 (100.00)	13 (100.00)		
Tibial plateau fracture accompanied by tibia	18	18 (100.00)	18 (100.00)		
Fracture of metaphysis or diaphysis					

Patella fracture	7	5 (71.43)	7 (100.00)	1.86 > 0.05	
Patellar transverse fracture	2	2 (100.00)	2 (100.00)		
Comminuted patellar fracture	3	3 (100.00)	3 (100.00)		
Longitudinal patella fracture	1	0 (0.00)	1 (100.00)		
Avulsion fracture of small patella	1	0 (0.00)	1 (100.00)		
Knee free body	3	0 (0.00)	3 (100.00)	9.00 < 0.01	

## Data Availability

The image data used to support the findings of this study have been deposited in the I Do Imaging (IDI) dataset (https://idoimaging.com/home).
